# Analysis of Prognostic Risk Factors of Endoscopic Submucosal Dissection (ESD) and Curative Resection of Gastrointestinal Neuroendocrine Neoplasms

**DOI:** 10.1155/2022/5248256

**Published:** 2022-07-08

**Authors:** Yuan Si, ChaoKang Huang, JingBin Yuan, XianHui Zhang, QingQiang He, ZhiJin Lin, Ling He, ZhongXin Liu

**Affiliations:** ^1^Endoscopic Center, XingTai People's Hospital, Xingtai 054001, China; ^2^Department of Pathology, XingTai People's Hospital, Xingtai 054001, China; ^3^Department of General Surgery, QuYang HengZhou Hospital, BaoDing 073100, China; ^4^Department of CT, XingTai People's Hospital, Xingtai 054001, China; ^5^Department of Gastrointestinal Surgery, XingTai People's Hospital, Xingtai 054001, China; ^6^Doctor Patient Office, XingTai People's Hospital, Xingtai 054001, China; ^7^Department of Otolaryngology, HeBei Eye Hospital, Xingtai 054001, China; ^8^Xingtai People's Hospital, No. 16, Hongxing Street, Xingtai, Hebei Province, China

## Abstract

**Objective:**

To explore the prognostic risk factors of ESD curative resection of gastrointestinal-neuroendocrine neoplasms (GI-NENs).

**Methods:**

A total of 97 patients treated with ESD successfully in our hospital were selected, their surgical site, size, number of resection lesions, operation time, intraoperative complications (such as bleeding and perforation), and treatment status were recorded, and the number of hemostatic clamps used after the postoperative follow-up results and the independent risk factors for ESD complications were obtained through the comparison between the noncomplication group and the ESD complication group using regression analysis.

**Results:**

A total of 97 patients with gastrointestinal neuroendocrine tumors were treated with ESD. 61 were males, 36 were females, the ratio of male to female was 1.7 : 1, onset age was 20–78 years old, and median onset age was 50 years old. In 81 cases, tumors were located in the stomach, 10 in the duodenum, and 6 in the rectum. A total of 103 lesions were detected by endoscopy, including 1 case with 2 sites in the stomach, 5 cases with 2 sites in the rectum, and the rest were single. The tumor diameter was 0.3 ∼ 2.5 cm, and the median diameter was 0.6 cm; there were 25 sites with a diameter less than 5 cm. There were 57 places with 10 mm, 16 places with 10–15 mm, and 5 places with >15 mm. All ESD operations were performed in one piece, with a total resection rate of 100%; 89.6% (60/67) of postoperative pathology showed negative basal, and 90.3% (56/62) showed negative resection margin, with a complete resection rate of 88.9% (48/54). ESD's operation time is 6 ∼ 66 min, and the median time is 18 min. During the operation, 5 cases had small amount of bleeding, 3 cases were perforated, 2 cases of delayed postoperative bleeding, 1 case of bleeding was caused by the patient's failure to follow the advice of the doctor to eat a large amount of solid food too early, and 1 case of delayed perforation (all recovered and discharged). ESD operation that bled, age, gender, and perforation location, pathological grade, pathological classification, tumor diameter, tumor surface, operation time, number of titanium clips, origin, echo uniformity, and echo level were statistically insignificant (*P* > 0.05). Postoperative bleeding was related to the operation time (*P*=0.017), but it was not an independent risk factor for postoperative bleeding (*P*=0.118; OR, 0.226; 95% CI, 0.035–1.461). 59 cases were followed up by endoscopy after the operation, and recurrence or no new tumors were found.

**Conclusion:**

ESD is an effective and safe treatment method for gastrointestinal neuroendocrine tumors with a diameter of 1-2 cm without invading the muscularis propria. The intraoperative complications seem to have little relationship with the patient; postoperative delayed bleeding is closely related to the ESD operation time but it is not an independent risk factor.

## 1. Introduction

Gastrointestinal-neuroendocrine neoplasms (GI-NENs) are a type of heterogeneous tumors originating from peptidergic neurons and neuroendocrine cells, which show obvious signs of slow growth from indolence and low-grade malignancy to high metastasis. A series of malignant biological behaviors [1] is distributed in various organs of the entire digestive tract. The incidence rate of neuroendocrine tumors was generally low in the past. But according to the data released by the National Cancer Institute (NCI) in 2004, the incidence rate of neuroendocrine tumors [2, 3] and neuroendocrine neoplasm (NEN) increased by 5 times in the past 30 years, from the original 1.09/10 to 5.25/10 million. The incidence rate of neuroendocrine tumors from the gastrointestinal tract is higher than that of other gastrointestinal cancers. GI-NENs have become the only gastrointestinal tract disease after colon cancer.

At present, the diagnosis of gastroenteric pancreatic-neuroendocrine neoplasm (GEP-NEN) mainly depends on clinical manifestations, tumor marker level, relevant imaging examinations (such as computerized tomography (CT) and magnetic resonance imaging (MRI) or digestive endoscopy), and “gold standard pathological examination.” According to the clinical manifestations of patients, gastroenteric pancreatic-neuroendocrine tumors (GEP-NET) can be divided into nonfunctional and functional tumors, most of which are nonfunctional tumors, which can be asymptomatic for many years. Most of them are accidentally found or manifested as compression symptoms caused by masses and signs of tumor metastasis. In this study, 154 patients with GEP-NEN showed typical carcinoid syndrome, accounting for only 1.3%, which is consistent with relevant literature reports at home and abroad [4]. Its clinical manifestations are very nonspecific, and it is difficult to accurately diagnose GEP-NEN by clinical manifestations alone. For patients with suspected GEP-NEN, corresponding tumor markers can be detected, such as insulinoma, peripheral blood insulin level, and gastrinoma, gastrin level. However, since such markers are only expressed in corresponding functional tumors, considering that most of the clinical findings are nonfunctional tumors, negative detection factors could not exclude the possibility of tumor existence. At present, sync onus (SYN) and comprehensive geriatric assessment (CGA) have been widely used as tumor markers for clinical detection of neuroendocrine tumors. Because sync onus (SYN) is widely expressed in GEP-NEN cells, it is diffusely positive and its sensitivity is high. The expression of CGA in GEP-NEN cells is related to the site of the disease. It is often weakly expressed in the lung and rectum, and its specificity is high, which is consistent with the results of this study. The total positivity rate of SYN is 93.9%, the total positivity rate of CGA is 38.5%, and the total positivity rate in the rectum is 28.6%. In combination with their advantages, it is recommended to detect SYN and CGA at the same time in the diagnosis of GEP-NEN patients.

At present, ESD treatment is the main choice for GEP-NEN tumors with tumor diameters less than 2 cm, no lymph node metastasis, infiltration depth not to the muscular propria, and well-differentiated GEP-NEN tumors [5]. However, sometimes the ESD treatment of GEP-NEN cannot be completely removed. So far, there are few reports on the risk factors of GEP-NEN ESD curative resection. Therefore, this research would explore this resection in detail.

The main purpose of this paper is how ESD is used for treating patients in their particular age durations. For this purpose, ESD has different procedures and methods. Using ESD methods, patients were treated with some ratio from male to female. Tumors with ESD were diagnosed, and the diameter and different complications were identified. Patients of this disease have different conditions due to their ages, and young age patients can have a better treatment than the old.

Section 1 discusses the introduction of the proposed work.  Section 2 defines the methodology for ESD patients and how to diagnose and treat them.  Section 3 describes the results using the ESD procedure.  Section 4 provides a discussion about diseases, treatments, and ratios of better results.  Section 5 discusses the conclusion of the whole work in the paper.

## 2. Materials and Methods

Participants were collected in our hospital from December 2019 to June 2021. Patients who successfully underwent ESD endoscopic resection and were pathologically diagnosed as gastrointestinal neuroendocrine tumors strictly implemented the inclusion and exclusion criteria. This study has been approved by the ethics committee of Xingtai People's Hospital and obtained the informed consent of patients. A total of 97 patients were enrolled, including 61 males and 36 females, aged 20–78 years old; the median age of onset was 50 years old.

### 2.1. Inclusion Criteria

1. Age >18 years old
2. The pathology department of our hospital diagnosed gastrointestinal neuroendocrine tumor
3. Treat patients with ESD

### 2.2. Exclusion Criteria

- Neuroendocrine tumors in other systems except for the digestive tract (such as urinary system, respiratory system, and reproductive system)
- The pathology department of our hospital has not diagnosed gastrointestinal neuroendocrine tumor
- Those who have ESD contraindications
- Exclude other fatal diseases

### 2.3. Equipment

Olympus UM-200 ultrasonic endoscopic system, UM-2R microprobe, OlympusQ260 or XQ260 electronic gastroscope, Olympus JF-240R electronic duodenoscope, Olympus JF-260R electronic duodenoscope, AGB high-frequency generator, HK knife, IT knife, injection needle, trap, hemostatic forceps, transparent cap, titanium clip, ventilator, and ECG monitoring were used.

### 2.4. ESD Preoperative

The lesion site and endoscopy results are recorded in detail according to the sex and age of the patient before surgery, and the blood biochemistry, coagulation function, electrocardiogram, chest X-ray, and lung function test are checked regularly. Possible complications such as substitution surgery, requirements and precautions for family members, intraoperative bleeding and perforation, late-onset bleeding, and late perforation should be informed to patients and families before surgery. Patients and their families can have a certain degree of understanding of the operation, eliminate their anxiety and fear, and sign the informed consent of the operation.

### 2.5. ESD Procedure

ESD operation steps are as follows [6]:

- *Marking.* The scope of the lesion was determined, and the spot electrocoagulation was marked on the outer edge of the lesion by about 5 mm
- *Submucosal Injection.* Submucosal injection (sodium hyaluronate injection) should be performed at the mark until the lesion is uniformly elevated
- *Incision of the Mucosa*. The lesion is incised at the lesion marker
- *Submucosal Dissection.* After the incision of the mucosa around the lesion, the lesion was exfoliated to the whole lesion
- *Treatment of Wounds.* The small vessels exposed on the wound surface were stopped by thermal hemostatic forceps, and the wound surface was closed by titanium clips
- *Specimen Processing*. The diseased tissue was smoothed and fixed on a thin plate with a pin and fixed with 10% neutral formalin

### 2.6. Postoperative Treatment

Postoperative fasting for 2 to 3 days, routine fluid replacement, using antibiotics and hemostatic drugs if perforation or bleeding occurs, observing abdominal symptoms and signs, and monitoring exhaust and defecation are done in postoperative treatment. All resected lesions were immersed in a 10% formalin solution and sent for pathological examination to determine the nature of lesions, the cutting edge of specimens, and whether tumor cells were involved in the base.

### 2.7. ESD Efficacy Evaluation

- Lump-sum resection: the lesion was a lump-sum resection under endoscopy
- Complete resection: at the pathological level, both horizontal and vertical resection margins of the whole specimen were negative
- Curative resection: complete resection with no or low risk of lymph node metastasis

### 2.8. Follow-Up Visit

All the enrolled patients were followed up with an endoscopic follow-up, which generally lasted from 1 to 3 months after ESD. The follow-up mainly included whether there were new lesions, whether the postoperative lesions were repaired, whether the levels were clear, and whether there were abnormal echo changes.

### 2.9. Statistical Analysis

The data were analyzed by SPSS18.0 statistical software, and the measurement data conforming to normal distribution were expressed as mean ± standard deviation; otherwise, the median was used as an expression, and the adoption rate or composition ratio of the series data was described. For qualitative data, when *n* ≥ 40 and all theoretical frequencies ≥5, Pearson chi-square test was used. Fisher's exact test was used for data that did not meet the chi-square test conditions. Univariate analysis was first used for patients with ESD complications. After confounding factors were excluded, logistic multifactor analysis was used to obtain independent risk factors. *P* < 0.05 was considered statistically significant.

## 3. Results

### 3.1. General Information

In this study, 97 patients with gastrointestinal-neuroendocrine tumors (GI-NET) were treated by ESD, including 61 males and 36 females, with a male to female ratio of 1.7 : 1. The onset age was 20–78 years, and the median onset age was 50 years.

### 3.2. Location and Diameter of the Tumor

Of the 97 GEP-NEN patients, 81 were located in the stomach, 10 in the duodenum, and 6 in the rectum. A total of 103 lesions were detected by endoscopy, including 2 lesions in the stomach in 1 case, 2 lesions in the rectum in 5 cases, and the rest were single. The diameter of the tumor was 0.3–2.5 cm, and the median diameter was 0.6 cm. There were 25 lesions with a diameter of <5 mm, 57 with a diameter of 5–10 mm, 16 with a diameter of 10–15 mm, and 5 with a diameter of >15 mm.

### 3.3. ESD Complications

ESD was successfully performed on all patients to remove the lesions; among which 2 cases underwent additional surgery due to the involvement and infiltration of tumor cells in the base as indicated by postoperative pathology. The operation time was 6–66 min, with a median time of 18 min. During the operation, 5 cases had a small amount of bleeding, which was stopped by hot biopsy forceps or titanium clips. There were 3 cases of perforation, 2 of which were clamped by intraoperative titanium clip, and the other one was not treated. There were 2 cases of delayed bleeding after the operation and 1 case of bleeding caused by eating a large amount of solid food prematurely without following the doctor's advice. All patients were cured by internal conservative treatment. Delayed perforation occurred in 1 case, which was clipped with a titanium clip under endoscopy.

### 3.4. Risk Factors in ESD Surgery

In this study, a total of 5 patients had intraoperative bleeding, 3 patients had intestinal perforation, and rectal bleeding was more than other parts of the bleeding. Therefore, the intestine can be divided into upper gastrointestinal tract and gastrointestinal division. Similarly, the pathological stage can be divided into G1 stage and G1 stage. The high degree of echo is divided into higher than normal group and lower than normal group. The origin can be divided into mucosal layer and mucosa. Then, we performed single-factor analysis on the suspected risk factors of ESD complications (age, sex, site, pathological grade, pathological classification, tumor diameter, tumor surface, operation time, number of titanium clips, origin, echo uniformity, and echo level) and intraoperative bleeding and perforation. After excluding confounding factors, factors with *P* < 0.05 were included in the binary logistic regression analysis model, and their independent risk factors were obtained. According to the analysis, age, gender, location, pathological grade, pathological classification, tumor diameter, tumor surface, operation time, number of titanium clips, source, echo uniformity, and echo level were not risked factors in EDS surgery, but the number of lesions may cause perforation.

According to the analysis in Tables 1 and 2, intraoperative bleeding and perforation had no significant correlation with age, sex, location, pathological grade, pathological classification, tumor diameter, tumor surface, operation time, number of titanium clips, origin, echo uniformity, and echo level.

### 3.5. Risk Factors after ESD

In this study, there were 2 cases of delayed postoperative bleeding and 1 case of delayed postoperative perforation. Considering that the incidence of postoperative perforation was very low <1%, this study focused on analyzing the risk factors of delayed postoperative bleeding. Suspicious risk factors for delayed bleeding were found in univariate analysis, including age, sex, location, pathological typing, tumor diameter, tumor surface, time of surgery, quantity, source, titanium forceps, echo uniformity, and echo height. And the operation time is related to postoperative bleeding. When included in logistic multifactor regression, it was found that it was not an independent risk factor for delayed postoperative bleeding. According to the analysis, age, gender, location, pathological grade, pathological classification, tumor diameter, tumor surface, operation time, number of titanium clips, source, echo uniformity, and echo level were not risk factors in EDS surgery (refer to Tables 3–5).

### 3.6. Postoperative Pathology

In this group, all ESD was removed in one block, and the removal rate of the whole block reached 100%. 89.6% (60/67) postoperative pathology suggested a negative base, 90.3% (56/62) suggested a negative margin, and the complete resection rate was 88.9% (48/54). Pathological results showed that 85 cases were *G*1 grade, 5 cases were *G*2 grade, and 7 cases were *G*3 grade. According to the pathological diagnosis consensus of gastrointestinal and pancreatic neuroendocrine tumors in China in 2011, there were 90 cases of NET and 7 cases of NEC.

### 3.7. Results Follow-Up

All the patients were followed up by endoscopy, of which 59 patients (52 *G*1, 4 *G*2, and 3 *G*3) were followed up by endoscopy. The endoscopic review showed that the resection sites of lesions were mostly recovered without new tumors or recurrence, and local mucosal thickening and clear hierarchical structure were most common.

## 4. Discussion

Currently, there is no unified treatment specification for the treatment of neuroendocrine tumors [6–12], and the existing diagnosis and treatment plan is a multidisciplinary comprehensive treatment based on individualization, which is divided into local stage and extensive stage according to whether the tumor patients have distant metastasis. For patients with extensive-stage GEP-NEN, the main treatment measures include surgical resection, endoscopic treatment, radiation interventional therapy, traditional chemotherapy, emerging biotherapy, and molecular targeted drug therapy. Regardless of whether GEP-NEN is functional or metastatic, surgical resection is the only cure [13], while surgery has its minimum surgical requirements [14]. Surgical treatment is an effective treatment that can improve the prognosis of patients, which is consistent with the results reported in many domestic and foreign literature [15]. The boundary between surgery and endoscopic treatment of gastrointestinal neuroendocrine tumors has always been controversial. Subsequently, in 2011, the National Comprehensive Cancer Network (NCCN) put forward the corresponding endoscopic and surgical diagnosis and treatment guidelines based on the tumor site [16–18].

Though some operation methods have reached a consensus, because of their low incidence, there is still considerable controversy in surgical methods and the lack of clinically credible and effective data to evaluate efficacy, so with the continuous development of endoscopic technology, compared with conventional surgery, endoscopic surgery has less trauma, fast recovery, and less cost, making more and more people choose endoscopic treatment. Since most gastrointestinal NENs tend to invade the submucosa [19], traditional endoscopic resection techniques often lead to positive resection margins, which makes it difficult to achieve complete resection and bring a second surgical blow to patients. Compared with traditional endoscopic resection techniques, ESD can achieve the whole resection of lesions with a larger diameter and more accurate pathological staging of specimens, thus achieving complete pathological resection, avoiding the shock of secondary surgery and reducing the economic burden on patients. Domestic scholars [20] treated 22 cases of gastrointestinal neuroendocrine tumors with the size of 0.2–1.5 cm by ESD, and the ESD whole resection rate reached 100%; the postoperative pathology indicated that the complete resection rate was 90.1% (20/22). No tumor recurrence or metastasis was observed during 6–24 months of postoperative follow-up. Some studies [21] used ESD to remove upper gastrointestinal neuroendocrine tumors with an average diameter of 0.9 cm, and all lesions were completely removed at one time, with a complete resection rate of 100%. Postoperative pathology indicated that the complete resection rate was 94.7% (18/19). In this group, the average lesion diameter was 0.67 ± 0.34 cm, the average operation time was 20.9 ± 110.8 min, and the ESD whole resection rate was 100%. 89.6% of postoperative pathology suggested a negative base, 90.3% suggested a negative edge, and the complete resection rate was 88.9%. No signs of local recurrence or distant metastasis were found in endoscopic follow-up 1–3 months after surgery. The effectiveness of ESD in the treatment of gastrointestinal neuroendocrine tumors was fully confirmed.

Bleeding and perforation are the most common complications of ESD treatment for GEP-NEN. Domestic reports reported that the incidence of intraoperative acute bleeding was 7.1% [19], and the incidence of intraoperative perforation was 4% [20]. However, the incidence of intraoperative bleeding during ESD in this study was 3.2%, and the incidence of intraoperative perforation was 1.9%, both lower than those reported in relevant literature [19, 20]. How to effectively prevent and treat intraoperative and postoperative wound bleeding is very important for the success of the surgery. Preoperative risk of bleeding should be fully evaluated, preoperative preparation should be made, and understanding and cooperation of patients should be obtained. Secondly, intraoperative bleeding may not only blur the intraoperative field of vision and affect the success of surgery but even in the case of a large amount of bleeding, it is difficult to stop bleeding under endoscopy, so ESD has to be terminated and surgical hemostasis has to be performed. Therefore, bleeding must be consciously prevented during ESD operation. For suspicious lesions, such as those found in the process of stripping blood vessels, in order to avoid the risk of bleeding, they can be clipped from the wall of the digestive tract by electrocautery or thermal biopsy forceps. Use norepinephrine (1 : 10 000) times to wash the wound, and remove the bleeding after endoscopic hemostasis. When necessary, we also can use mucosa protectant (medical glue) covering the wound or the use of hemostatic clamp (titanium clip blood vessels). Our study found that patients with intraoperative bleeding with age, sex, disease, pathologic stage, and no significant correlation between pathological type consider ESD to be difficult and complex operation and at the same time needs an assistant to cooperate. Intraoperative bleeding may be related to the operator's operating experience, skill proficiency, and medical cooperation. Perforation is another major complication of ESD. Titanium clips can be used to close small perforations. Perforation is closed with nylon rope suture clips, gastrointestinal decompression tubes are used after surgery, fasting for several days is done, antibiotics are supplemented to prevent infection, intravenous nutritional support is established, and re-operation can generally be avoided.

A definitive diagnosis of GEP-NEN requires a pathological diagnosis. Compared with other similar studies at home and abroad [22], NEN had a higher survival rate. The main consideration was that it was compared with other digestive tract malignancies; NEN progressed slowly and had a better prognosis, and some tumors could be completely resected. Univariate survival analysis showed that age, site, distant metastasis, and pathological grade were closely related. The younger the patient, the better the prognosis. The lower the pathological grade, the better the prognosis. The prognosis of patients without distant metastasis was better than that of patients with distant metastasis. Patients with tumors located in the lower gastrointestinal tract have a better prognosis than patients with the upper gastrointestinal tract, which is consistent with some foreign literature reports [23].

## 5. Conclusion

Gastrointestinal neuroendocrine tumors, as potential malignant tumors of the digestive system, have a low incidence rate, which can occur anywhere in the digestive tract and lack specific clinical manifestations. These factors have led to the difficulty of diagnosing the disease in the past. With the increasing incidence rate of the disease and the improvement of the level of diagnosis, GEP-NEN has gradually entered our field of vision. Surgical resection has been the preferred treatment for this disease. It has been popular. In recent years, with the development of endoscopic technology, ESD has been used as an effective and safe treatment for GEP-NEN. However, because of the low incidence rate of gastrointestinal neuroendocrine tumors, the sample size of this study is small, and patients need to choose bias. The research results of large samples are further confirmed.

## Figures and Tables

**Table 1:** Risk factor analysis of qualitative data during ESD.

Factors	Bleeding	No bleeding	Perforated	Unbroken	*X* ^2^		*P*	
					Bleeding	Perforated	Bleeding	Perforated
Sex						0.220	1.000	0.606
Male	3	58	1	60				
Female	2	34	2	34				
Parts							0.588	1.000
Upper gastrointestinal tract	0	17	0	17				
The digestive tract	5	81	3	83				
Pathological grade							1.000	0.313
*G*1	5	86	2	89				
Non-*G*1	0	12	1	11				
Pathological classification							1.000	0.300
NET	5	91	2	94				
NEC	0	12	1	11				
Tumor surface							1.000	1.000
Smooth	4	75	3	76				
Erosion	1	21	0	22				
Origin							0.237	1.000
The mucous membrane layer	1	4	0	5				
Nonmucosal layer	4	88	3	89				
Echo uniformity							1.000	0.286
Uniformity	1	17	1	17				
Intermingle	2	43	0	45				
Echo height							1.000	1.000
Higher than normal group	0	10	0	10				
Lower than normal group	5	82	3	84				

**Table 2:** Risk factors analysis of quantitative data during ESD.

Factors	Bleeding	No bleeding	Perforated	Unbroken	*Z*		*P*	
					Bleeding	Perforated	Bleeding	Perforated
Age	46	50	47	51	−0.449	−1.105	0.653	0.269
Diameter	0.5	0.6	0.6	0.6	−0.067	−0.797	0.946	0.426
Operation time	21	18	22	18	−1.675	−1.189	0.094	0.234
Number of lesions	1	1	1	1	−0.590	−1.959	0.555	0.050
Number of titanium clips	4	4	5	4	−0.216	−0.212	0.829	0.832

**Table 3:** Risk factor analysis of qualitative data of delayed bleeding in ESD.

Factors	Bleeding	No bleeding	*X* ^2^	*P*
Sex				0.528
Male	2	59		
Female	0	36		
Parts				1.000
Upper gastrointestinal tract	0	17		
The digestive tract	2	84		
Pathological grade				0.220
*G*1	1	90		
*Non*-*G*1	1	11		
Pathological classification				0.211
NET	1	95		
NEC	1	6		
The tumor surface				1.000
Smooth	2	77		
Erosion	0	22		
Origin				1.000
The mucous membrane layer	0	5		
Nonmucosal layer	2	90		
Echo uniformity				0.286
Uniformity	1	17		
Intermingle	0	45		
Echo height				1.000
Higher than normal group	0	10		
Lower than normal group	2	85		

**Table 4:** Risk factor analysis of quantitative data of delayed bleeding in ESD.

Factors	Bleeding	No bleeding	*Z*	*P*
Age	51	50	−0.038	0.970
Diameter	0.7	0.6	−0.223	0.824
Operation time	1	1	−0.367	0.714
Number of lesions	2	4	−1.638	0.101
Number of titanium clips	7	18	−2.390	0.017

**Table 5:** Logistic regression analysis of delayed bleeding in ESD.

Factors	B	Wald	Sig	OR	95% CI	
					Lower	Upper
Operation time	−1.486	2.439	0.118	0.226	0.035	1.461

## Data Availability

The datasets used and analyzed during the current study are available from the corresponding author upon reasonable request.

## References

[1] Oberndorfer S. (1907). Karzinoide Tumoren des Dunndarms. *Frankfurter Zeitschrift für Pathologie*.

[2] Öberg K. (2010). 1. Neuroendocrine tumors (NETs): historical overview and epidemiology. *Tumori Journal*.

[3] Yao J. C., Hassan M., Phan A. (2008). One hundred years after “carcinoid”: epidemiology of and prognostic factors for neuroendocrine tumors in 35,825 cases in the United States. *Journal of Clinical Oncology*.

[4] Tsikitis V. L., Wertheim B. C., Guerrero M. A. (2012). Trends of incidence and survival of gastrointestinal neuroendocrine tumors in the United States: a seer analysis. *Journal of Cancer*.

[5] Hauso O., Gustafsson B. I., Kidd M. (2008). Neuroendocrine tumor epidemiology. *Cancer*.

[6] Godwin J. D. (1975). Carcinoid TumorsAn analysis of 2837 cases. *Cancer*.

[7] Cho M. Y., Cho M.-Y., Sohn J. H. (2013). Proposal for a standardized pathology report of gastroenteropancreatic neuroendocrine tumors: prognostic significance of pathological parameters. *Korean Journal of Pathology*.

[8] Delle Fave G., Kwekkeboom D. J., Van Cutsem E. (2012). ENETS Consensus Guidelines for the management of patients with gastroduodenal neoplasms. *Neuroendocrinology*.

[9] Falconi M., Bartsch D. K., Eriksson B. (2012). ENETS Consensus Guidelines for the management of patients with digestive neuroendocrine neoplasms of the digestive system: well-differentiated pancreatic non-functioning tumors. *Neuroendocrinology*.

[10] Caplin M., Sundin A., Nillson O. (2012). ENETS Consensus Guidelines for the management of patients with digestive neuroendocrine neoplasms: colorectal neuroendocrine neoplasms. *Neuroendocrinology*.

[11] Pavel M., Baudin E., Couvelard A. (2012). ENETS Consensus Guidelines for the management of patients with liver and other distant metastases from neuroendocrine neoplasms of foregut, midgut, hindgut, and unknown primary. *Neuroendocrinology*.

[12] Salazar R., Wiedenmann B., Rindi G., Ruszniewski P. (2012). ENETS 2011 consensus guidelines for the management of patients with digestive neuroendocrine tumors: an update. *Neuroendocrinology*.

[13] Jensen R. T., Cadiot G., Brandi M. L. (2012). ENETS Consensus Guidelines for the management of patients with digestive neuroendocrine neoplasms: functional pancreatic endocrine tumor syndromes. *Neuroendocrinology*.

[14] Pape U.-F., Perren A., Niederle B. (2012). ENETS Consensus Guidelines for the management of patients with neuroendocrine neoplasms from the jejuno-ileum and the appendix including goblet cell carcinomas. *Neuroendocrinology*.

[15] Berge T., Linell F. (2009). Carcinoid tumours. *Acta Pathologica et Microbiologica Scandinavica Section A Pathology*.

[16] Yucel B., Babacan N. A., Kacan T. (2013). Survival analysis and prognostic factors for neuroendocrine tumors in Turkey. *Asian Pacific Journal of Cancer Prevention*.

[17] Sekiguchi M., Sekine S., Sakamoto T. (2015). Excellent prognosis following endoscopic resection of patients with rectal neuroendocrine tumors despite the frequent presence of lymphovascular invasion. *Journal of Gastroenterology*.

[18] Ishido K., Tanabe S., Higuchi K. (2010). Clinicopathological evaluation of duodenal well-differentiated endocrine tumors. *World Journal of Gastroenterology*.

[19] Kulke M. H., Benson A. B., Bergsland E. (2012). Neuroendocrine tumors. *Journal of the National Comprehensive Cancer Network*.

[20] Mullen J. T., Wang H., Yao J. C. (2005). Carcinoid tumors of the duodenum. *Surgery*.

[21] Yoshikane H., Tsukamoto Y., Niwa Y. (1993). Carcinoid tumors of the gastrointestinal tract: evaluation with endoscopic ultrasonography. *Gastrointestinal Endoscopy*.

[22] Oda I., Saito D., Tada M. (2006). A multicenter retrospective study of endoscopic resection for early gastric cancer. *Gastric Cancer*.

[23] Modlin I. M., Lye K. D., Kidd M. (2003). A 5-decade analysis of 13,715 carcinoid tumors. *Cancer*.

